RETRACTED

# Associations of Changes in Intestinal Flora and Inflammatory Factors with Prognosis of Patients with Esophageal Cancer

**DOI:** 10.1155/2022/2426301

**Published:** 2022-03-27

**Authors:** Cheng Wu, Ming Wang, Qing Zhou, Hui Shi

**Affiliations:** Department of Gastroenterology, The Second Medical Center and National Clinical Research Center for Geriatric Diseases, Chinese PLA General Hospital, Beijing 100853, China

## Abstract

This study aims to explore the associations of changes in intestinal flora and inflammatory factors with the prognosis of patients with esophageal cancer (EC). A total of 40 EC patients treated and 40 normal people who underwent gastroscopy and CT examination for gastrointestinal discomfort during the same period were selected as the participants of the study. The endotoxin level, colonization ability of intestinal flora, and distribution of intestinal flora (*Bifidobacterium*, *Lactobacillus*, *Escherichia coli*, and *Enterococcus*) were compared between the two groups. The levels of inflammatory factors interleukin-6 (IL-6), high-sensitivity C-reactive protein (hs-CRP), and tumor necrosis factor-*α* (TNF-*α*) were also compared between the two groups. All participants were followed up for 3 years, and the associations of survival time with colonization ability of intestinal flora and changes in hs-CRP were analyzed. Finally, the univariate and multivariate logistic regression analyses were performed for related factors affecting the survival time of EC patients. In the observation group, the endotoxin level was significantly higher (*P* < 0.05), the colonization ability of intestinal flora was significantly weaker (*P* < 0.05), the levels of *Bifidobacterium* and *Lactobacillus* were obviously lower (*P* < 0.05), and the levels of *Escherichia coli* and *Enterococcus* were obviously higher than those in the normal group (*P* < 0.05). Besides, the observation group had abnormal and evidently higher levels of IL-6, hs-CRP, and TNF-*α* than the normal group (*P* < 0.05). The survival time was positively correlated with the colonization ability of intestinal flora (*P* < 0.05), but negatively correlated with the changes in hs-CRP (*P* < 0.05). Moreover, the increased level of endotoxin, weakened colonization ability of intestinal flora, abnormal distribution of intestinal flora, and elevated levels of inflammatory factors were all related and independent risk factors affecting the survival time of EC patients. In EC patients, the endotoxin level markedly rises, the colonization ability of intestinal flora declines, and there are intestinal flora disorders and enhanced inflammatory response. With the decline in colonization ability of intestinal flora and the increase of inflammatory response, the survival time of EC patients will be shortened.

RETRACTED

## 1. Introduction

Esophageal cancer (EC) is the 8th most common type of cancers worldwide and constitutes the 6th leading cause of cancer deaths, characterized with high mortality rate and poor prognosis at time of diagnosis and variability based on geographic location [1]. The occurrence of EC is related to a variety of factors, such as diet, genetics, and living environment. There are no obvious clinical manifestations in the early stage, so EC has been mostly in the middle and late stages when diagnosed, often leading to poor prognosis. EC is mainly treated with radical operation, combined with comprehensive interventions, such as postoperative chemoradiotherapy and biotherapy [2]. With the constant advance in medical technology and treatment in recent years, the survival time and prognosis of EC patients have been greatly improved. However, operation and postoperative chemoradiotherapy cause great impact on the patient's body [3].

Due to the characteristics of EC after onset, patients suffer from long-term difficulty in eating, varying degrees of malnutrition, low immunity, and enhanced inflammatory response [4]. In addition, the surgical trauma is large, and the vagal nerve trunk needs cutting off during operation, thus leading to redistribution of blood flow. The patients still cannot eat via the digestive tract, especially the mouth, in the short term after operation. As a result, the dysfunction will occur in gastrointestinal motility, absorption, and barrier, and inflammatory factors will be released [5]. As the body's most important organ related to nutrient absorption, the gastrointestinal tract plays a distinctly important role in the nutritional support of the human body, especially that of patients with malignant tumors. Moreover, the gastrointestinal tract is highly valuable in the body's immunoregulation and inflammatory responses [6]. In order to better improve the intestinal function of EC patients, this study aims to explore the changes in intestinal flora and inflammatory factors in patients and analyze the associations between such changes and prognosis of patients. It is now reported as follows.

## 2. Materials and Methods

### 2.1. General Data

A total of 40 EC patients and 40 normal people who underwent gastroscopy and CT examination for gastrointestinal discomfort during the same period (normal group) were selected as the participants of the study. EC patients were diagnosed via pathological biopsy during the operation, and they signed the informed consent before enrollment. This study was approved by the Ethics Committee of Chinese PLA General Hospital. Inclusion criteria were as follows: participants aged 18–50 years old, those with normal mental conditions and regular life, and those treated with operation after onset. Exclusion criteria were as follows: participants with mental disease, immune system disease, or other digestive tract diseases, those who took drugs affecting intestinal flora distribution within 1 month before enrollment, those with an estimated survival time of less than 3 months, or those with tumor cachexia. In the observation group, there were 26 males and 14 females aged 18–50 years old with an average of (45.6 ± 3.7) years old. The clinical symptoms lasted for 1 week to 3 months, with an average of (1.3 ± 0.2) months. The body mass index (BMI) at the time of enrollment was 20–25, with an average of (21.9 ± 1.3). In terms of the educational level, there were 33 cases of senior high school and above and 7 cases below senior high school. In the normal group, there were 25 males and 15 females aged 18–50 years old with an average of (45.5 ± 3.7) years old. The clinical symptoms lasted for 1 week to 3 months, with an average of (1.4 ± 0.2) months. The BMI at the time of enrollment was 20–25, with an average of (21.8 ± 1.3). In terms of the educational level, there were 32 cases of senior high school and above and 8 cases below senior high school. There were no statistically significant differences in gender, age, duration of clinical symptoms, BMI at the time of enrollment, and educational level between the two groups (*P* > 0.05).

RETRACTED

### 2.2. Methods

Midsegment fresh feces (0.5 g) naturally defecated last time before operation were obtained from EC patients, and 0.5 g of fresh feces naturally defecated first time in the morning of the day after enrollment was obtained from healthy people. The samples were placed into the MGIEasy sample collection kit and immediately sent for detection. Then, 4.5 mL of diluent was added, and 10 *μ*L of samples was inoculated into 4 selective media of *Bifidobacterium*, *Lactobacillus*, *Escherichia coli*, and *Enterococcus*, followed by incubation at 37°C for 24–48 h. Then, the related intestinal bacteria were counted and identified based on the number of viable bacteria on the plate. At the same time, 5 mL of cubital venous blood was drawn in the morning of the day after enrollment in both groups, and blood biochemical indexes were detected via enzyme-linked immunosorbent assay (ELISA).

### 2.3. Observation Indexes

The endotoxin level, colonization ability of intestinal flora, and distribution of intestinal flora (*Bifidobacterium*, *Lactobacillus*, *Escherichia coli*, and *Enterococcus*) were compared between the two groups. The levels of inflammatory factors interleukin-6 (IL-6), high-sensitivity C-reactive protein (hs-CRP), and tumor necrosis factor-*α* (TNF-*α*) were also compared between the two groups. All participants were followed up for 3 years, and the associations of survival time with colonization ability of intestinal flora and changes in hs-CRP were analyzed. Besides, the univariate and multivariate logistic regression analyses were performed for related factors affecting the survival time of EC patients.

RETRACTED

### 2.4. Evaluation Criteria

The colonization ability of intestinal flora was evaluated by *Bifidobacterium*/*Escherichia coli* (B/*E*) ratio (normal value >1). The intestinal endotoxin level was detected via the azoic developing process (normal value < 0.1 EU/mL). Next, *Bifidobacterium*, *Lactobacillus*, *Escherichia coli*, and *Enterococcus* were detected in this study. The reference value is 0.37–0.46 ng/L for IL-6, 0–100 mg/L for hs-CRP, and 5–100 ng/L for TNF-*α*.

### 2.5. Statistical Analysis

Statistical Product and Service Solutions (SPSS) 13.0 software (SPSS Inc., Chicago, IL, USA) was used for statistical processing. Measurement data were expressed as mean ± standard deviation (‾*χ* ± *s*). The *t*-test was performed for the comparison of means between two groups, and the *χ*^2^ test was used for the comparison of rates between two groups. The univariate and multivariate logistic regression analyses were performed for factors affecting the survival time of EC patients, and Pearson correlation analysis was also adopted. *P* < 0.05 suggested the statistically significant difference.

## 3. Results

### 3.1. Comparison of Endotoxin Level and Colonization Ability of Intestinal Flora between the Two Groups

In the observation group, the endotoxin level was significantly higher (*P* < 0.05), and the colonization ability of intestinal flora was significantly weaker than those in the normal group (*P* < 0.05) (Table 1).

### 3.2. Comparison of Distribution of Intestinal Flora between the Two Groups

In the observation group, the levels of *Bifidobacterium* and *Lactobacillus* were obviously lower (*P* < 0.05), and the levels of *Escherichia coli* and *Enterococcus* were obviously higher than those in the normal group (*P* < 0.05) (Table 2).

### 3.3. Comparison of Inflammatory Factor Levels between the Two Groups

Compared with the normal group, patients in the observation group exhibited evidently higher levels of IL-6, hs-CRP, and TNF-*α* (*P* < 0.05) (Table 3).

### 3.4. Correlation Analysis of Survival Time with Colonization Ability of Intestinal Flora and Changes in hs-CRP

The survival time was positively correlated with the colonization ability of intestinal flora (*r* = 0.9215, *P* < 0.001), but negatively correlated with the changes in hs-CRP (*r* = −0.9453, *P* < 0.001) (Figures 1 and 2).

RETRACTED

### 3.5. Univariate Analysis of Factors Affecting the Survival Time of EC Patients

It was found that the increased level of endotoxin, weakened colonization ability of intestinal flora, abnormal distribution of intestinal flora, and elevated levels of inflammatory factors were all related risk factors affecting the survival time of EC patients (Table 4).

### 3.6. Multivariate Analysis of Factors Affecting the Survival Time of EC Patients

The results revealed that the increased level of endotoxin, weakened colonization ability of intestinal flora, abnormal distribution of intestinal flora, and elevated levels of inflammatory factors were all independent risk factors affecting the survival time of EC patients (Table 5).

## 4. Discussion

Surgical intervention combined with postoperative chemoradiotherapy is the first choice in the treatment of EC. However, most of EC patients will suffer from severe malnutrition due to difficulty in swallowing and consumptive changes in the body caused by malignant tumor [7–9]. Meanwhile, due to surgical trauma, inability of early oral feeding, and stress stimulation, the body remains in a hypermetabolic and hypercatabolic state for a long time, and diarrhea, regurgitation, and emptying disorder may occur after operation, thereby further increasing the burden and causing intestinal dysfunction and intestinal flora disorders [10]. In the case of intestinal flora disorders, there will be obviously more pathogenic bacteria and massive release of endotoxin in patients with malignant tumors, thus affecting the normal function of intestinal flora. Moreover, the metabolites produced can also act on susceptibility genes, leading to immune response and accelerating growth and division of malignant tumor cells [11]. In addition, the elevated levels of inflammatory factors in the body are also important causes of development and early distant metastasis of malignant tumors [12].

The normal intestinal flora plays an important role in the body, which has a mutually symbiotic relation with the human body. It improves digestive function, assists food digestion, promotes nutrient absorption, boosts the body's immunity via secreting immune factors, and inhibits the colonization of pathogenic bacteria, thereby positively influencing human health [13]. Under normal conditions, *Escherichia coli* and *Enterococcus* are dominated in the surface layer, facultative anaerobic bacteria in the middle layer, and *Bifidobacterium* and *Lactobacillus* in the deep layer in the human body [14]. *Bifidobacterium* and *Lactobacillus* can bind tightly to the specific receptors of intestinal mucosal epithelial cells to form the biological barrier fixing the bacterial membrane, thereby resisting the invasion of pathogenic bacteria [15]. Abnormalities in the composition or distribution of the above bacteria indicate intestinal flora disorders [16]. There is a certain correlation between the occurrence and development of EC and the intestinal flora disorders [17]. Intestinal flora disorders can enhance the intestinal mucosal inflammatory response and increase the release of inflammatory factors, thus causing esophageal mucosal epithelial damage and abnormality in repair mechanism, ultimately resulting in tumors [18]. In addition, some bacterial metabolites and/or enzymes can exert a cytotoxic effect on esophageal epithelial cells, leading to incomplete metaplasia of esophageal mucous epithelium and malignant tumors [19]. Meanwhile, intestinal flora disorders will also bring about changes in the dietary structure and digestive ability of human body, thus causing malnutrition and reducing immunity. Then, the tumor burden further becomes larger, and early cachexia occurs, affecting the survival time of patients [20].

RETRACTED

In this study, according to the comparison of the endotoxin level and colonization ability of intestinal flora between the two groups, it was found that the endotoxin level was significantly higher, and the colonization ability of intestinal flora was significantly weaker in the observation group than those in the normal group. It can be seen that EC patients have a markedly higher level of endotoxin and markedly weakened colonization ability of intestinal flora. Then, it was observed that the levels of *Bifidobacterium* and *Lactobacillus* were obviously lower, and the levels of *Escherichia coli* and *Enterococcus* were obviously higher in the observation group than those in the normal group. The above results suggest that EC patients have obvious disorders of intestinal flora, characterized by the decline in the levels of *Bifidobacterium* and *Lactobacillus* and increase in the levels of *Escherichia coli* and *Enterococcus*. At the same time, the levels of inflammatory factors were compared between the two groups. The results showed that the observation group had abnormal and evidently higher levels of IL-6, hs-CRP, and TNF-*α* than the normal group, indicating that there are evidently more inflammatory factors and enhanced inflammatory response in EC patients. Besides, the correlation analysis results revealed that the survival time was positively correlated with the colonization ability of intestinal flora, but negatively correlated with the changes in hs-CRP. The above findings demonstrate that with the decline in colonization ability of intestinal flora and the increase of inflammatory response, the survival time of EC patients will be negatively impacted and shortened. Finally, it was confirmed that the increased level of endotoxin, weakened colonization ability of intestinal flora, abnormal distribution of intestinal flora, and elevated levels of inflammatory factors were all related and independent risk factors affecting the survival time of EC patients.

RETRACTED

## 5. Conclusions

In conclusion, in EC patients, the endotoxin level markedly rises, the colonization ability of intestinal flora declines, and there are intestinal flora disorders and enhanced inflammatory response. With the decline in colonization ability of intestinal flora and the increase of inflammatory response, the survival time of EC patients will be shortened.

## Figures and Tables

**Figure 1:** Correlation analysis between survival time and colonization ability of intestinal flora.

**Figure 2:** Correlation analysis between survival time and changes in hs-CRP.

**Table 1:** Comparison of endotoxin level and colonization ability of intestinal flora between the two groups.

	Endotoxin level (EU/mL)	Colonization ability of intestinal flora
Normal group	0.8 ± 0.1	1.4 ± 0.2
Observation group	1.3 ± 0.2	0.7 ± 0.1
*t*	14.142	19.799
*P*	<0.001	<0.001

**Table 2:** Comparison of distribution of intestinal flora between the two groups (LgN/g).

	*Bifidobacterium*	*Lactobacillus*	*Escherichia coli*	*Enterococcus*
Normal group	9.2 ± 0.5	8.0 ± 0.6	9.0 ± 0.4	7.1 ± 0.3
Observation group	7.5 ± 0.3	5.8 ± 0.3	10.5 ± 0.6	8.6 ± 0.5
*t*	18.439	20.742	13.156	16.270
*P*	<0.001	<0.001	<0.001	<0.001

**Table 3:** Comparison of inflammatory factor levels between the two groups.

	IL-6 (ng/L)	hs-CRP (mg/L)	TNF-*α* (ng/L)
Normal group	0.3 ± 0.1	61.3 ± 10.5	60.1 ± 5.3
Observation group	1.3 ± 0.2	138.9 ± 23.3	156.6 ± 32.3
*t*	28.284	19.204	18.646
*P*	<0.001	<0.001	<0.001

**Table 4:** Univariate analysis of factors affecting the survival time of EC patients.

		EC	No EC	*χ* ^2^	*P*
Endotoxin level	Increase	35	1	55.000	<0.001
	Normal	5	39		
Colonization ability of intestinal flora	Decrease	38	4	31.746	<0.001
	Normal	2	36		
Distribution of intestinal flora	Abnormal	36	6	42.155	<0.001
	Normal	4	34		
Inflammatory factors	Increase	34	10	57.836	<0.001
	Normal	6	30		

**Table 5:** Multivariate analysis of factors affecting the survival time of EC patients.

	*β*	W	SE	*P*	OR	95% CI
Increased level of endotoxin	1.12	6.39	5.51	<0.001	3.08	1.76–5.34
Weakened colonization ability of intestinal flora	2.35	9.93	0.46	0.01	2.81	1.21–4.41
Abnormal distribution of intestinal flora	1.83	4.83	0.58	0.04	1.97	1.03–7.46
Elevated levels of inflammatory factors	0.55	0.72	0.65	0.39	0.58	0.16–2.06

RETRACTED

## Data Availability

The datasets used and analyzed during the current study are available from the corresponding author upon request.
